# Changes of DCE‐MRI Parameters in Patients with Rheumatoid Arthritis before and after Therapy and Their Value for the Efficacy Evaluation of Patients

**DOI:** 10.1155/2021/6848359

**Published:** 2021-10-18

**Authors:** Danguo Chen, Shengquan He

**Affiliations:** ^1^Department of Imaging, Ningbo No. 6 Hospital, Ningbo 315040, China; ^2^Department of Imaging, 906 Hospital of the Joint Logistics Support Force of the Chinese People's Liberation Army, Ningbo 315000, China

## Abstract

**Objective:**

To explore the changes of dynamic contrast-enhanced magnetic resonance imaging (DCE-MRI) parameters in patients with rheumatoid arthritis (RA) before and after therapy and their value for the efficacy evaluation of patients.

**Methods:**

Totally, 90 patients with RA confirmed in our hospital between January 2018 and January 2020 were enrolled. All of them were examined with a Siemens Magnetom Avanto 1.5T imaging system, and data about the rate of enhancement in early stage (REE) and steep slope maximum (SSmax) were obtained. Then, the disease activity score in 28 joints (DAS-28), REE, and SSmax were analyzed, and the associations of SSmax and REE with erythrocyte sedimentation rate (ESR), C-reactive protein (CRP), and DAS-28 were investigated. Additionally, the patients were assigned to the acute-stage group and the chronic-stage group according to their time-signal intensity curves after therapy, and the two groups were compared in SSmax, REE, ESR, CRP, and DAS-28. Corresponding receiver operating characteristic (ROC) curves were drawn for the analysis of potential markers for efficacy improvement in patients.

**Results:**

After therapy, REE, SSmax, ESR, DAS-28, and CRP in the synovium of all patients declined greatly (all *P* < 0.05), with higher levels observed in the acute-stage group than those in the chronic-stage group (all *P* < 0.05). SSmax and REE of patients were positively bound up with their ESR, CRP, and DAS-28 (all *P* < 0.05). Additionally, according to ROC curve-based analysis, both SSmax and REE can be adopted as biological indexes for distinguishing between patients at the acute phase from those at the chronic stage, and joint detection of them can boost the sensitivity of DAS-28.

**Conclusion:**

The SSmax and REE levels in RA patients after treatment were significantly decreased, and the levels in patients in the chronic phase were lower than those in patients in the acute phase. SSmax and REE are highly expressed in RA patients, and the combined detection can enhance the value of DAS-28 in the assessment of RA, and it is worthy of clinical promotion.

## 1. Introduction

Rheumatoid arthritis (RA) is a common autoimmune disease, which is characterized by chronic synovitis and mainly damages synovial joints [1, 2]. According to statistics, its incidence in China ranges between 0.2% and 0.4%. RA can cause inflammation, joint injury, deformity, and disability [3]. Its most frequent initial manifestation is inflammatory arthritis involving facet joints in the hand, and damaged frequently used hand joints (metacarpophalangeal joint, proximal interphalangeal joint, and wrist joint) are one crucial reason for adults to lose their self-care ability [4, 5]. With the emergence of antirheumatic drugs in the past decades, RA has achieved a better prognosis [6], but early diagnosis and early therapy are the key to reducing its disability rate [7].

RA is recurrent, so patients with it should visit doctors regularly to have evaluation of activity and treatment effect [8]. 28-joint disease activity score (DAS-28) is an evaluation method based on erythrocyte sedimentation rate (ESR) and clinical manifestations, which is often used for clinical evaluation of RA patients [9] and clinical manifestations [10]. However, the method is carried out mainly based on patients' clinical symptoms, laboratory examination, and wrist X-ray results, so it has main limitations in revealing the condition of affected joints and the accuracy of disease progress evaluation [11]. In addition, due to subjective factors, DSA-28 may lead to subjective bias in disease evaluation [12].

According to recent studies at home and abroad [13, 14], magnetic resonance imaging (MRI), especially dynamic contrast‐enhanced MRI (DCE-MRI), is of profound clinical value for the early diagnosis and progress of RA because of its high sensitivity to various pathological changes of affected joints. DCE-MRI can display the proliferation of the synovial pannus in patients with RA. Parameters such as early enhancement rate (REE) and maximum steep slope (SSmax) calculated from the time-signal intensity curve can quantify the severity of synovitis, which is a research focus on the early diagnosis of RA and the determination of disease activity. The pathological basis of perfusion effect is the number of blood vessels and their permeability in the inflammatory synovial membrane as well as the necessary extracellular space. That is to say, the changes of signal intensity on DCE-MRI perfusion imaging mainly depend on the vascular density in the diseased tissue and the amount of the contrast agent entering the extracellular space of the tissue. The degree of enhancement of the lesion depends on the degree of vascularization of the lesion, the permeability of the vascular contrast agent, and the extracellular fluid volume. During the first passage of the contrast agent, the capillary bed of the lesion filled with the contrast agent was mainly located in the blood vessel, but it was rarely located outside the vessel. The concentration gradient inside and outside the vessel was the largest, and the change of signal strength was rarely affected by diffusion factors, mainly due to the change of the dose of the contrast agent inside the vessel. Therefore, REE and SSmax evaluating the early changes in signal strength at this time could reflect the blood perfusion rate of the lesion and indirectly reflect the microvascular distribution of the tissue, thereby reflecting the pathological changes of the inflammatory synovial membrane. However, relevant literature studies on the value of DCE-MRI in evaluating the clinical efficacy on RA are scant. Accordingly, this study was conducted for exploring the changes of DCE-MRI parameters in patients with RA before and after therapy and their value for the efficacy evaluation of patients, with the aim of offering a more effective examination means to the clinical efficacy evaluation of RA.

## 2. Materials and Methods

### 2.1. Clinical Data

Totally, 90 patients with RA confirmed in our hospital between January 2018 and January 2020 were enrolled, including 19 males and 71 females between 30 and 67 years old, with a mean age of 49.6 ± 10.7 years. All the patients presented with swelling and pain in the hands and wrist joints as the chief complaint, and there was no positive finding on hand X-ray films. The course of the disease was from 2 to 24 months. This study was performed with approval of the Ethics Committee of our hospital, and informed consent forms were signed by all patients after being apprised of the study. The inclusion criteria were as follows: patients meeting the RA diagnostic criteria jointly proposed by the American College of Rheumatology (ACR) and European League Against Rheumatism (EULAR) in 2010 [15], patients confirmed with RA at the first diagnosis in our hospital, and patients at the acute stage. In this study, disease course ≤1 year and no obvious bone changes on the X-ray plain film were taken as the judgment criteria of early RA meantime. The exclusion criteria were as follows: patients without detailed case data, patients who had received antirheumatic drugs were used before enrollment in this study, patients intolerant of this treatment plan, and those reluctant to cooperate with follow-up and treatment.

### 2.2. Therapeutic Regimen

All patients were given methotrexate and leflunomide meantime. Specifically, the patient was injected with methotrexate (Jiangsu Hengrui Pharmaceutical Co., Ltd., State Food and Drug Administration (SFDA) approval no. H32026443) at an initial dose of 7.5 mg per week, and the dosage was gradually increased to 12.5 mg per week, once a week. The patient was also required to orally take 25 mg leflunomide (Suzhou Changzheng-Cinkate Pharmaceutical Co., Ltd., SFDA no. 20060034), twice a day, for 3 months.

### 2.3. MRI Examination Mode

In this study, MRI examination was conducted with a Siemens Magnetom Avanto 1.5T imaging system. Specifically, the patient was given routine MRI scan in a prone position, with palms down, under the following sequences: for coronal fast spin echo (FSE) T1WI: TR: 500 ms, TE: 11 ms, ETL = 7, slice thickness: 3 mm, slice spacing: 0.3 mm, scanning field of view: 240 mm × 240 mm, and matrix: 358 × 358; for coronary fat-suppressed FSE T2WI: TR: 3,000 ms, TE: 30 ms, ETL: 7 mm, slice thickness: 3 mm, slice spacing: 0.3 mm, scanning field of view: 240 mm × 240 mm, and matrix: 240 × 240; for transverse FSE T2WI: TR: 4,180 ms, TE: 83 ms, ETL = 7, slice thickness: 3.5 mm, slice spacing: 0.35 mm, scanning field of view: 120 mm × 120 mm, and matrix: 268 × 268. The plain scan images were evaluated, and the lesions were accurately located, followed by dynamic enhanced scanning. The patient was injected with contrast agent Gd-DTPA by the intravenous bolus injection technique with a high-pressure syringe at an injection rate of 2.5 ml/s and a dose of 0.1 mmol/kg, and then 15 mL isotonic saline was injected at the same flow rate to flush the pipeline. With an acquisition time of 10 s, 35 phases were acquired during 350 s. After the dynamic enhanced scanning, the patient was given conventional enhanced T1WI scanning on coronal and transverse planes.

### 2.4. Image Analyses

The data obtained after scanning were analyzed in the Siemens Syngo View workstation and processed. The region of interest (ROI) was drawn in the most prominent synovial hyperplasia, on which the ROI time-signal intensity curve was acquired. In addition, REE and SSmax were calculated.

### 2.5. DAS-28 Calculations

The clinical observation indexes including the number of joint swelling, the number of joint tenderness, and laboratory test data were collected. According to the clinical observation index DAS-28 = 0.56 × √TJC + 0.28 × √SJC + 0.7 × IN (ESR) + 0.014 × PG (1.3), where TJC is the painful joint count, SJC is the swollen joint count, ESR is the erythrocyte sedimentation rate, and PG is the overall health assessment of the patient.

### 2.6. Outcome Measures

The primary outcome measures were as follows: the changes of REE, SSmax, ESR, C-reactive protein (CRP), and DAS-28 before and after therapy were evaluated, and the association of REE and SSmax with ESR, CRP, and DAS-28 was analyzed.

The secondary outcome measures were as follows: the patients were assigned to the acute-stage group and the chronic-stage group according to their ROI time-signal intensity curves after therapy, and the two groups were compared in SSmax, REE, ESR, CRP, and DAS-28 after therapy. Corresponding receiver operating characteristic (ROC) curves were drawn for the analysis of potential markers for efficacy improvement in patients.

### 2.7. Statistical Analyses

This study adopted SPSS 24.0 for statistical analyses of the data and GraphPad 8 for visualization of the data into corresponding figures. Count data were analyzed via the chi-square test, and intergroup comparisons of measurement data (mean ± SD) were conducted by the independent-sample *T*-test and their intragroup comparisons by the paired *t*-test. ROC curves were adopted for the evaluation value analysis of each index in patients with acute or chronic RA, and Pearson's test was adopted for the association analysis of REE and SSmax with ESR, CRP, and DAS-28. *P* < 0.05 denotes a notable difference.

## 3. Results

### 3.1. Imaging Characteristics

A total of 90 patients with RA were included according to inclusion and exclusion criteria. Synovial hyperplasia and pannus formation were present in the articular surface of the wrist in all patients, with blurring of the involved facet joint spaces and swelling of the surrounding soft tissues (Figure 1). 60 of them showed signs of carpal bone marrow edema with the heterogeneous bone signal, and mixed hypointense signal could be seen on T1WI. 40 cases showed bone erosion, and the involved facet joints were not smooth or there were small sheets of bone erosion.

### 3.2. Changes of Indexes before and after Therapy

We evaluated the changes of SSmax, REE, ESR, CRP, and DAS-28 of patients before and after therapy and found notable decreases of them in the patients after therapy (all *P* < 0.01, Figure 2).

### 3.3. Correlation Analysis of SSmax and REE with ESR, CRP, and DAS-28

We also found correlations of SSmax and REE with ESR, CRP, and DAS-28. As displayed in Figure 3, ESR, CRP, and DAS-28 were all positively bound up with SSmax and REE (all *P* < 0.01).

### 3.4. Changes of Various Indexes in Patients at the Acute Stage and Those at the Chronic Stage

In this study, the patients were classified into fast-rising type (acute stage, *n* = 55) and slow-rising type (chronic phase, *n* = 35) according to their perfusion curves. We compared the changes of SSmax, REE, ESR, CRP, and DAS-28 between the two kinds of patients and found notably lower levels in patients at the chronic stage than those at the acute stage (all *P* < 0.05, Figure 4).

### 3.5. Evaluation Value of Each Index in Acute and Chronic Stages of Patients

In this study, we also analyzed the evaluation value of each index in acute and chronic stages of patients with RA.  Figure 5 demonstrates a high clinical value of SSmax, REE, ESR, CRP, and DAS-28 in the evaluation of acute and chronic RA (Table 1). DAS-28 score is a frequently adopted evaluation index for patients with RA. Lastly, we analyzed the evaluation value of DAS-28 combined with SSmax or REE in acute and chronic RA.  Figure 6 reveals that, with SSmax or REE, DAS-28 can deliver a higher value in evaluating acute and chronic RA (Table 2).

## 4. Discussion

Pathological changes of RA mainly include synovitis, pannus formation, synovial hyperplasia, and erosion of the articular cartilage and subchondral bone. Acute RA is mainly characterized by exudative and inflammatory cell infiltration, joint distortion in the later stage, and even loss of limb movement function [16]. The so-called active period and remission period of RA are essentially the manifestation of synovitis in acute and stable periods, respectively [17]. At present, ESR, CRP, and DAS-28 are mostly used to evaluate the inflammatory activity of RA, but the results of laboratory indexes are often biased due to various factors [18]. DAS-28 is an accurate method to evaluate RA activity, but it is limited because of its inability to reflect the microcirculation information inside the lesion.

MRI can provide high-resolution, multidirectional, multiparameter, and multisequence images for soft tissue, so its value in the early diagnosis of RA has been clinically recognized because it can help to find pathological changes of early RA, such as synovitis, pannus, bone marrow edema, bone erosion, and tenosynovitis [19]. However, due to the complex grading process of the MRI system, its clinical application is limited. As the medical level and medical instruments advance continuously, DCE-MRI has demonstrated great advantages in the quantitative analysis of pathological changes of RA [20]. According to prior research [21], DCE-MRI has confirmed the ability of synovial enhancement rate to quantify the activity degree of RA synovitis. In addition, one other study has revealed the ability of DCE-MRI in evaluating hand erosive osteoarthritis and psoriatic arthritis [22]. In our study, we evaluated the changes of DCE-MRI parameters and ESR, CRP, and DAS-28 of patients with RA before and after therapy and found notable decreases of SSmax, REE, ESR, CRP, and DAS-28 in patients after therapy. Through correlation analysis, we also found that SSmax and REE were positively correlated with ESR, CRP, and DAS-28, which indicated that SSmax and REE might become the observation indexes of rheumatoid arthritis development [23]. DCE-MRI parameters were calculated according to ROI time-signal intensity curves. The formation of the posterior pannus after RA leads to thicker microvessel density, incomplete microvascular wall, and larger interstitial cavity. The small-molecule intravascular contrast agent can leak into the enlarged extracellular space rapidly through the damaged vascular wall, which causes the ROI time-signal intensity curve to be mainly of fast-rising plateau type, which has the characteristics of steep ascending branch, entering the plateau period after reaching the peak value, and the peak time is the shortest [24].

RA is chronic and recurrent, so it is necessary to adjust its treatment regimen in time [25]. As the application of hormones and nonsteroidal anti-inflammatory drugs, clinical symptoms or inflammatory indicators are mitigated sensitively [26]. In our study, ESR and CRP changed significantly before and after treatment, but for other patients with comorbidity, their specificity will decrease because of influences of comorbidity [27]. In our study, the patients were classified into acute-stage patients and chronic-stage patients according to their perfusion curves, and they were compared in indexes in different periods after therapy. It was found that chronic-stage patients showed lower levels of SSmax, REE, ESR, CRP, and DAS-28 than acute-stage patients. Additionally, according to ROC curve-based analysis, the area under the curve (AUC) of each index was lower than 0.7, and that of both SSmax and REE was greater than 0.8. The results imply that both SSmax and REE can serve as potential indexes to evaluate acute and chronic phases of patients. DAS-28 is a commonly used index for the clinical evaluation of RA. Its sensitivity in this study is not high, but its specificity in RA evaluation reached 100.00% in this study. Therefore, it is of far-reaching value to improve the sensitivity of DAS-28 in assessing rheumatoid arthritis. At the end of our study, we drew curves of DAS-28 combined with SSmax and DAS-28 combined with REE and found the AUCs of the two combinations were 0.957 and 0.966, respectively, and their combination strongly boosted the sensitivity of DAS-28. It follows from the results that the joint detection of SSmax, REE, and DAS-28 can improve the evaluation of patients' disease severity.

In our study, we found high expressions of SSmax and REE in rheumatoid arthritis patients and their ability to improve the sensitivity of DAS-28 in the evaluation of rheumatoid arthritis. However, this study still has some limitations. First of all, this study has not included the control group, so whether there are differences in SSmax and REE between patients with RA and healthy individuals needs further analysis. Secondly, the period of this study is short, and a large number of samples have been removed according to the inclusion and exclusion criteria. Therefore, we hope to collect more samples and add a control group in the follow-up study to further analyze the SSmax and REE values of RA patients.

To sum up, SSmax and REE presented high expression in patients with RA, and joint detection of them can boost the value of DAS-28 in RA evaluation, so their joint detection is worthy of clinical promotion.

## Figures and Tables

**Figure 1:** Wrist imaging characteristics of patients with RA. (a) A DCE-MRI image of the healthy wrist. (b) A DCE-MRI image of RA patients' wrist.

**Figure 2:** Changes of SSmax, REE, ESR, CRP, and DAS-28 scores in patients before and after therapy. (a) Changes of SSmax before and after therapy according to DCE-MRI. (b) Changes of REE before and after therapy according to DCE-MRI. (c) Changes of ESR before and after therapy according to the results detected by the Westergren method. (d) Changes of CRP before and after therapy according to the results detected by ELISA. (e) Changes of DAS-28 of patients before and after therapy. ^*∗∗*^*P* < 0.01 and ^*∗∗∗*^*P* < 0.001.

**Figure 3:** Correlation analysis of SSmax and REE with ESR, CRP, and DAS-28. (a) Analysis of the correlation between SSmax and ESR by Pearson's test. (b) Analysis of the correlation between SSmax and CRP by Pearson's test. (c) Analysis of the correlation between SSmax and DAS-28 by Pearson's test. (d) Analysis of the correlation between REE and ESR by Pearson's test. (e) Analysis of the correlation between REE and CRP by Pearson's test. (f) Analysis of the correlation between REE and DAS-28 by Pearson's test.

**Figure 4:** Changes of various indexes in patients at the acute stage and those at the chronic stage. (a) Changes of SSmax in patients at the acute stage and those at the chronic stage according to DCE-MRI. (b) Changes of REE in patients at the acute stage and those at the chronic stage according to DCE-MRI. (c) Changes of ESR in patients at the acute stage and those at the chronic stage according to results obtained by the Westergren method. (d) Changes of CRP in patients at the acute stage and those at the chronic stage according to results obtained by ELISA. (e) Changes of DAS-28 scores in patients at the acute stage and those at the chronic stage after therapy. ^*∗*^*P* < 0.05 and ^*∗∗*^*P* < 0.01.

**Figure 5:** ROC curves of SSmax, REE, ESR, CRP, and DAS-28 in the evaluation of acute and chronic RA. (a) Evaluation value of SSmax in acute and chronic RA according to ROC curve-based analysis. (b) Evaluation value of REE in acute and chronic RA according to ROC curve-based analysis. (c) Evaluation value of ESR in acute and chronic RA according to ROC curve-based analysis. (d) Evaluation value of CRP in acute and chronic RA according to ROC curve-based analysis. (e) Evaluation value of DAS-28 in acute and chronic RA according to ROC curve-based analysis.

**Figure 6:** Evaluation value of DAS-28 combined with SSmax or REE in acute and chronic RA. (a) Evaluation value of SSmax combined with DAS-28 in acute and chronic RA according to ROC curve-based analysis. (b) Evaluation value of REE combined with DAS-28 in acute and chronic RA according to ROC curve-based analysis.

**Table 1:** ROC curve parameters of SSmax, REE, ESR, CRP, and DAS-28 in evaluation of acute and chronic RA.

Index	AUC	95 CI%	Specificity	Sensitivity	Youden's index	Cutoff
SSmax	0.860	0.784–0.936	91.42	72.72	64.15	>4.295
REE	0.850	0.772–0.929	94.28	69.09	63.37	>3.270
ESR	0.765	0.669–0.861	85.71	61.81	47.53	>29.23
CRP	0.782	0.689–0.875	100.00	54.54	54.54	>21.42
DAS-28	0.748	0.650–0.846	100.00	45.45	45.45	>4.115

**Table 2:** DAS-28 combined with SSmax or REE in acute and chronic RA.

Index	AUC	95 CI%	Specificity	Sensitivity	Youden's index	Cutoff
SSmax and DAS-28	0.957	0.902–1.000	94.28	96.36	90.64	>0.501
REE and DAS-28	0.966	0.924–1.000	100.00	94.54	94.54	>0.625

## Data Availability

The data used and analyzed are available from the corresponding author upon reasonable request.
